# Evaluation of Metal Ion Concentration in Hard Tissues of Teeth in Residents of Central Poland

**DOI:** 10.1155/2017/6419709

**Published:** 2017-01-19

**Authors:** Piotr Wychowanski, Konrad Malkiewicz

**Affiliations:** ^1^Department of Oral Surgery, Medical University of Warsaw, Warsaw, Poland; ^2^Department of Orthodontics, Medical University of Warsaw, Warsaw, Poland

## Abstract

*Objectives.* The aim of the study was an assessment of the content of trace elements in enamel and dentin of teeth extracted in patients residing in urban and agricultural areas of Poland.* Methods.* The study included 30 generally healthy patients with retained third molars. 65 samples of enamel and dentin from individuals living in urban areas and 85 samples of enamel and dentin from individuals living in agricultural areas were prepared. The content of manganese, lead, cadmium, and chromium in the studied enamel and dentin samples from retained teeth was determined by Graphite Furnace Atomic Absorption Spectrometry. In the process of statistical hypothesis testing, the level of significance was assumed at *α* = 0.05.* Results.* A comparative analysis of the data showed that enamel and dentin of inhabitants of industrialized areas contain significantly higher amounts of lead and cadmium than hard tissues of teeth in residents of agricultural areas and comparable amounts of manganese and chromium.* Significance.* It appears that hard tissues of retained teeth may constitute valuable material for assessment of long-term environmental exposure to metal ions. The study confirms that the risk of exposure to heavy metals depends on the place of residence and environmental pollution.

## 1. Introduction

Metals are elements widely found in the environment. They form natural deposits around the world and are widely used in many areas of life. Some of those elements, such as iron and copper, are essential for life and proper functioning of the body, playing an important role in metabolic processes. Other elements do not play a significant role in physiological processes; moreover, they can contribute to defects in organs as well as individual tissues, impair their function, and induce a broad spectrum of diseases in the mechanism of acute poisoning resulting from intensive supply and of chronic exposure to relatively low doses [1]. Due to their harmful biological effects, special attention is devoted to exposure and mechanisms of adverse action of trace elements such as lead, cadmium, manganese, and chromium on the human organism.

These metals can originate from industrial pollution including dust, sewage, combustion products of fossil fuels, paints and varnishes, tobacco smoke, everyday objects, and food contaminated with the above [2, 3]. The presence of metallic elements has been observed in all parts of the ecosystem including the water, the atmosphere, the soil, and plants.

Lead is commonly used in industry for production of batteries, cables, wires, or bearings; it may be a component of paint or varnish. It is also present in solders widely used in the electronics industry. Until recently, lead compounds which are contained in gasoline were one of the main sources of systemic exposure to the harmful element [4] and although in Europe and the United States unleaded fuel is commonly used, certain developing countries have not as yet introduced necessary regulations to eliminate the element from the production processes in the petrochemical industry.

Exposure to lead and its compounds during both the prenatal and postnatal periods causes damage to the nervous system and disorders of renal function or gastrointestinal tract. This element can also cause damage to liver or components of the hematopoietic system [5]. In the case of increased concentration in the body, lead can be responsible for developmental disorders of the nervous system manifested by behavioral changes, in both children and adults [6, 7]. Lead has been classified as a potentially carcinogenic element [8] in the International Agency for Research on Cancer classification.

Cadmium is widely used in production processes of alloys including copper, zinc, and iron. It is also used in production of highly specialized electronic products such as microchips or motherboards of computers [9]. Therefore, it is a component of the so-called “e-waste,” whose disposal is often carried out improperly or is associated with release of many biologically harmful chemicals into the environment.

According to IARC classification, cadmium is considered a dangerous carcinogenic factor [8]. It is also assumed that exposure to the element causes damage to kidneys and developmental disorders of the skeleton [10, 11]. Increased supply of cadmium during both prenatal and postnatal development can affect the development of the nervous system and consequently be the cause of concentration disorders and hyperactivity in children [12, 13]. It is also believed to have negative impact on spermatogenesis [14]. Apart from workers employed in heavy or electronic industries, also tobacco smokers and people in their vicinity are particularly exposed to the pathogenic effects of cadmium.

Manganese is used in the metallurgical, chemical, and ceramic industries. It is also used in the manufacture of dyes, pesticides, and fertilizers. Similar to lead and cadmium, it can be potentially harmful to health in case of increased supply. High exposure to manganese can cause damage to the respiratory system [15]. This element has a particularly negative effect on maturation and function of the nervous system [15, 16].

Chromium, similar to lead and cadmium, is classified by IARC as a factor inducing development of cancer [8]. It is used in production of dyes, tannins, and cements. This element is present in anticorrosion coatings obtained in the process of galvanization. Exposure to chromium can cause skin lesions and disorders of the respiratory and digestive systems [17]. It also demonstrated mutagenic and embryotoxic action [18–20].

The increasing pollution of the environment associated with the development of civilization makes us vulnerable to the rising supply of heavy metals.

Monitoring the content of substances potentially dangerous to health in the human body is essential for assessing health hazards for individuals and populations being at risk of exposure to heavy metals. Evaluation of the content of biologically harmful trace elements in the body may therefore be the starting point for the implementation of preventive and curative measures for the exposed individuals, as well as contributing to introduction of system solutions limiting the emission of heavy metals into the environment and minimizing the effects of occupational exposure.

Several methods for determination of metals in biological tissues are currently available, for example, inductively Coupled Plasma- (ICP-) Mass Spectrometry (MS) [21] or Ion Chromatography [22, 23]. In the present study the authors applied the Graphite Furnace Atomic Absorption Spectrometry (GFAAS) method, a sensitive and specific technique, which has been used by many clinical chemistry laboratories to determine the presence of trace metals in physiological fluids and in tissues.

## 2. Aim

The aim of the study was a comparative assessment of the content of trace elements in enamel and dentin of teeth extracted for surgical indications in patients residing in urban and agricultural areas of central Poland.

## 3. Material and Methods

The study included generally healthy patients living in the Mazowieckie province. Patients were qualified on the basis of the dental surgery health questionnaire and the clinical history card. Individuals working in heavy or chemical industries as well as tobacco smokers were excluded, as well as patients systematically taking vitamin-mineral preparations. A total of thirty generally healthy subjects were qualified, aged 26 to 37 years with fully impacted third molars, which had no contact with the environment of the oral cavity. Thirteen of the enrolled individuals, including seven females and six males, lived in the Warsaw metropolitan area, while seventeen patients, including nine females and eight males, inhabited rural areas of the Mazowieckie province.

Each subject underwent surgical extraction of one of retained third molars. The procedures were performed under local anesthesia and the teeth intended for analysis were removed entirely. In total 30 teeth were extracted from which samples of enamel and dentin were obtained for assessment in the study, five for each tissue type. Immediately after the treatment, the teeth were cleaned from soft tissue residue and rinsed with distilled water and then with HPLC-grade water. From the prepared teeth, samples of enamel and dentin were prepared with diamond drill bits under microscope control, in order to perform quantitative analysis of identified elements, independently for both fractions. After mechanical division of a tested tooth, enamel and dentin samples were left for 24 hours in 30% solution of H_2_O_2_ to remove organic contaminants, then washed with distilled water and high purity HPLC-grade water, dried at 80°C, and finally ground. Sixty-five samples of enamel and dentin from individuals living in the city of Warsaw were prepared (five for each of the thirteen patients), as well as eighty-five samples of enamel and dentin from individuals living in agricultural areas of the Mazowieckie province (five for each of the seventeen patients). The obtained material was analyzed for the content of lead, cadmium, manganese, and chromium, separately for enamel and dentin of the assessed teeth.

The assay method used for the content of manganese, lead, cadmium, and chromium in the samples of enamel and dentin of the retained teeth was Graphite Furnace Atomic Absorption Spectrometry (GFAAS). The obtained values are given in micrograms per one gram of assessed sample.

In all cases, a variant of the calibration curve was used, whose range matched the concentration of an assessed element in the analyzed material. The detection threshold of the elements identified in the study ranged from 0.02 to 0.05 *μ*g/l. The study used Avanta Ultra atomic absorption spectrometer by GBC, with PAL 4000 automatic sample dispenser and graphite furnace.

## 4. Ethical Considerations

The study was approved by the Bioethical Committee of the Medical University of Warsaw (approval number KB 219/2016). Participation in the study was voluntary, and the patients were informed about its course and assumptions and granted the right to withdraw from the study. Confidentiality of patient data with respect to the results was ensured by assigning numerical codes to samples of biological material subjected to analysis.

## 5. Methods of Statistical Analysis

Statistical analysis was performed using STATISTICA 8.0 software.

In the process of hypothesis testing the level of significance was assumed at *α* = 0.05.

When the choice was determined by the researcher, conclusions were based on the two-sided critical region.

For each continuous variable, basic statistics were calculated: number (*n*), the arithmetic mean ($\overset{-}{X}$), standard deviation (SD), median, minimum and maximum values, and indicators of skewness and kurtosis.

In the analysis of means for independent variables, in the case of two-point grouping variable, Student's *t*-tests or Cochran-Cox tests were used, depending on the result of *F* test with which the assumption of equal variances was tested. In the case of a three-point grouping variable, ANOVA was used. The assumption of equal variances was tested with Brown-Forsythe tests. Newman-Keuls tests were used as post hoc tests. For the analysis of dependent variables, Student's *t*-tests were used.

Correlation analysis was based on Pearson and Spearman correlation coefficients. The significance of correlation coefficients was tested with corresponding Student's *t*-test.

In regression analysis a linear regression model was used. The parameters were estimated by the least squares method.

## 6. Results

The average concentration of cadmium in the enamel of impacted teeth of residents of agricultural areas of Mazowieckie province equaled 0.015 *μ*g/g and was significantly lower (*p* ≤ 0.05) than the concentration of cadmium in the samples of enamel of Warsaw metropolitan area residents, averaging 0.020 *μ*g/g.

The dentin of teeth extracted from residents of rural communities contained an average of 0.025 *μ*g/g of cadmium, whereas dentin in Warsaw residents demonstrated an average of 0.046 *μ*g/g of this element. These concentrations were statistically significantly different (*p* ≤ 0.05).

The average concentration of cadmium in the hard tissues of teeth in residents of agricultural areas was 0.020 *μ*g/g, while in the case of hard tissue obtained from the inhabitants of urban areas it was significantly higher, at 0.033 *μ*g/g.

Average concentrations of cadmium in dentin and enamel are shown in Table 1.

The average concentrations of chromium in the enamel of teeth in residents of agricultural and urban areas remained at the same level and equaled 0.510 *μ*g/g.

The average content of the element in the dentin tissue obtained from residents of both populations also assumed the same values and amounted to 0.640 *μ*g/g. The average concentration of chromium in hard tissues of the impacted and extracted teeth was 0.575 *μ*g/g, regardless of the individuals' place of residence.

Average concentrations of chromium in dentin and enamel are shown in Table 2.

The average concentration of manganese in hard tissues of retained teeth in residents of agricultural areas in Mazowieckie province was 0.485 *μ*g/g: the enamel contained an average of 0.639 *μ*g/g and dentin contained 0.320 *μ*g/g of this element. The average concentration of manganese in hard tissues of teeth obtained from residents of Warsaw metropolitan area was 0.485 *μ*g/g: enamel contained on average 0.640 *μ*g/g, while for dentine the value was 0.320 *μ*g/g. As in the case of chromium content, manganese also demonstrated no differences in the concentrations of the element in the evaluated hard tissues of teeth in both populations of patients.

Average concentrations of manganese in dentin and enamel are shown in Table 3.

The average concentration of lead in the enamel of teeth in residents of agricultural areas averaged 1.208 *μ*g/g and was significantly (*p* ≤ 0.05) lower than the concentration in the tissue obtained from the inhabitants of urban areas, which amounted to 1.655 *μ*g/g. The lead content in the dentine of teeth obtained from the rural residents did not differ significantly (*p* ≥ 0.05) from the content of the element in the tissue of teeth of urban residents. These values averaged, respectively, 2.110 *μ*g/g and 2.315 *μ*g/g. In total, the hard tissues of retained teeth in residents of agricultural areas demonstrated significantly lower (*p* ≤ 0.05) lead concentration at 1.659 *μ*g/g, compared with enamel and dentine samples obtained from urban residents, which on average contained 1,985 *μ*g/g of the element.

Average concentrations of lead in dentin and enamel are shown in Table 4.

## 7. Discussion

Lead, cadmium, manganese, and chromium are deposited in tissues and cause pathogenic action not only on individual organs but also on the whole body. In order to assess the concentration of trace elements in the organism, body fluids such as blood and urine are analyzed, as well as samples biopsied from individual organs including liver or kidney, bone fragments, and teeth [24].

Samples of blood and urine are easy to obtain. Their analysis, however, provides information only about recent and short-term exposure to harmful chemical substances. In this way the level of heavy metals in individual tissues is not detected either, which constitutes information about long-term exposure. Collecting biopsy samples from solid organs and bone tissue is technically difficult and is not a method used for screening.

The material, which is commonly available and at the same time easy to obtain, is hard tissue of teeth, that is, enamel and dentin. Because they are not as extensively metabolised as bone tissue [25], they constitute a reservoir of heavy metal ions, whose concentration informs us about the effects of long-term exposure to harmful elements in the context of health risk assessment. It is assumed that the level of metals observed in tissues of teeth correlates with their presence in the bloodstream, especially in the context of long-term exposure [26]. Deciduous teeth, which are lost naturally, constitute relatively easily accessible material for analysis. However, due to the processes of forming and mineralization of the enamel and dentin during the prenatal and postnatal periods, they provide information about exposure to heavy metals of fetuses and young children [27, 28]. It should also be noted that results of tissue analysis of deciduous teeth do not have to be one hundred percent reliable because of the placenta partially protecting fetuses against transmission of harmful elements from the mother's body and because children are usually protected against harmful environmental influences, which in adults can be associated with occupational exposure. Determining the concentration of harmful elements in the bodies of adults by analyzing the enamel and dentin refers to permanent teeth. Their development falls on the postnatal period and lasts—in the case of third molars—until about 20 years of age. Impacted teeth seem to constitute particularly valuable material for research, having no contact with the environment of the oral cavity even after the eruption period. They can provide research material on the basis of which we can assess the degree of prolonged exposure to heavy metals in adults.

The results of the present study indicate that hard tissues of evaluated impacted teeth contained significantly more lead and cadmium in the case of samples from the inhabitants of large urban areas than enamel and dentin of teeth extracted from the rural residents.

No studies in available literature describe the concentration of trace elements in enamel and dentin of the Polish population. Available literature describing studies from other parts of the world contains reports confirming the above observation.

A study by Costa de Almeida et al. [29], assessing the concentration of lead in the surface layers of tooth enamel, demonstrated significantly higher concentration of the element in samples from urban residents compared to samples of enamel in inhabitants of nonindustrialized areas. Similar observations were made by other authors [30, 31].

Prodana et al. [32] evaluated the concentration of cadmium in enamel and dentin of deciduous teeth of children living in industrialized and rural areas. The results reported by the authors from Romania indicate that the potentially harmful biological element was present in greater amounts in hard tissues of teeth of children living in highly industrialized areas at risk of environmental contamination.

Similar observations were made by authors from Spain [33] evaluating the relationship between place of residence and cadmium content in hard tissue of deciduous teeth, who confirmed the existence of a positive correlation between high environmental contamination and a higher concentration of a pathogenic element in enamel and dentin.

The above observations support the thesis, as reflected in the results of the present study, that concentration of lead and cadmium in hard tissues of teeth depends on the place of residence of the population whose samples were evaluated, and it is correlated with environmental pollution.

A different opinion was presented in the publication by Maah et al. [34]. The study evaluated cadmium content in hard tissues of permanent teeth extracted from residents of two different regions of Malaysia. The authors did not confirm the existence of a positive correlation between the concentration of the element and the place of residence; however, they noted that such a link exists in the case of cigarette smoking and suggested that the lack of significant differences could result from similar diet of patients living in both regions of the country included in the study.

Because the present study excluded patients declaring tobacco smoking, which is a major source of exposure to cadmium, it seems that the results are more meaningful in the context of exposure to the element resulting from environmental contamination.

In the available literature there are no publications correlating the concentration of manganese and chromium in hard tissues of teeth with the degree of environmental contamination. The study did not report the existence of any relationship between concentrations of these elements in enamel and dentin on one hand and the place of residence of the patients from whom tissue samples were collected on the other hand.

The reason for the lack of such correlation may be exclusion from the study of people working in heavy and chemical industries, which are predisposing factors for exposure to chromium and manganese in the context of occupational risk.

The literature provides relatively numerous reports assessing the concentration of metallic elements in hard tissues of deciduous teeth [29–40]. Unfortunately, the results published therein cannot be directly referred to the observations made in the present study because those publications evaluate the content of potentially harmful elements in deciduous teeth or, less frequently, in permanent teeth exposed to the oral environment.

Third molars, which were used in the present study, constitute a slightly different material for physicochemical analysis. It should be noted that they appear in the oral environment relatively late or remain in the bone tissue as impacted teeth, so they do not accumulate in themselves or accumulate in relatively small quantities, elements which have direct contact with their surface. Most often they are not exposed to masticatory forces; therefore, tooth crowns, which are used for samples to be analyzed, are not mechanically damaged. In the case of analysis of tissue composition of retained teeth, the influence of the external environment is eliminated, that is, drinks, food, temperature differences, and action of cariogenic microorganisms. Analyzed samples of third molars provide information about the influence of the external environment during the period from about seven to about eighteen years of age, when their buds are formed and mineralized. Therefore, they constitute a kind of 10-year carrier of data about diet, health, and human exposure to the effects of trace elements found in the external environment.

In a study by Liu et al. [41] the authors evaluated the content of phosphorus, calcium, strontium, barium, and lead in the enamel and dentine of third molars extracted for surgical indications. In their study the researchers from Taiwan used both impacted teeth and teeth in contact with the environment of the oral cavity of patients aged 17 to 68 years. The results presented by Liu et al. [41] allow identification of age groups 20–25 years and 25–30 years in the assessed population, roughly corresponding to the age group of patients evaluated in the present study.

The average concentration of lead in enamel of teeth in patients from Taiwan aged 20–25 years was about 0.53 *μ*g/g, while in the group of 26–30-year-olds it equaled about 0.77 *μ*g/g. The concentration of the element in the dentine of third molars evaluated by Liu et al. was 1.07 *μ*g/g and 0.7 *μ*g/g, respectively, for the studied age groups and it was significantly higher than its content in the enamel tissue.

The results of the present study confirm the reports by researchers from Taiwan [41] according to whom enamel has a lower potential to accumulate lead ions than dentine, which can be associated both with the period of development, during which both tissues are formed as well as with their chemical composition.

The results obtained by the authors from Taiwan [41] describing a lower concentration of lead in the hard tissues of teeth, compared to the concentrations noted in the present study, may indicate different environmental exposure to this element, which is potentially harmful to health with respect to both populations. Another reason for differences in results in terms of quantity could be the use of different analytical methods.

## 8. Conclusion

Despite an ever-expanding knowledge about the negative influence of heavy metal ions on the body, we still do not know the whole spectrum of their negative impact on human health. There is no doubt, however, that the risk of exposure to potentially harmful biological trace elements should be minimized, not only in particularly exposed occupational groups, but also in whole populations. One of the components of health risk assessment is monitoring the content of harmful elements in the body. In contrast to hair or body fluids, impacted teeth, obtained as a result of routine dental surgical procedures, seem to constitute extremely valuable material that allows quantitative and qualitative assessment of long-term exposure of patients to chemicals potentially dangerous to health.

The results of the present study confirm that the risk of exposure to heavy metals depends on the place of residence and is associated with environmental pollution.

In order to ensure the highest reliability of further studies, it is necessary to include possibly the largest group of patients, strictly observing the inclusion/exclusion criteria.

## Figures and Tables

**Table 1:** Average concentration of cadmium in hard tissues of impacted teeth (*μ*g/g).

Tissue	Enamel			Dentin			Total		
Place of residence	Concentration (*μ*g/g)	SD	*α* = 0.05	Concentration (*μ*g/g)	SD	*α* = 0.05	Concentration (*μ*g/g)	SD	*α* = 0.05
Urban	0.020	0.002	*p* = 0.0001	0.046	0.008	*p* = 0.0001	0.033	0.005	*p* = 0.0001
Rural	0.015	0.002		0.025	0.009		0.020	0.005	

**Table 2:** Average concentration of chromium in hard tissues of impacted teeth (*μ*g/g).

Tissue	Enamel			Dentin			Total		
Place of residence	Concentration (*μ*g/g)	SD	*α* = 0.05	Concentration (*μ*g/g)	SD	*α* = 0.05	Concentration (*μ*g/g)	SD	*α* = 0.05
Urban	0.510	0.188	*p* > 0.05	0.640	0.1723	*p* > 0.05	0.575	0.180	*p* > 0.05
Rural	0.510	0.188		0.640	0.1723		0.575	0.180	

**Table 3:** Average concentration of manganese in hard tissues of impacted teeth (*μ*g/g).

Tissue	Enamel			Dentin			Total		
Place of residence	Concentration (*μ*g/g)	SD	*α* = 0.05	Concentration (*μ*g/g)	SD	*α* = 0.05	Concentration (*μ*g/g)	SD	*α* = 0.05
Urban	0.640	0.117	*p* > 0.05	0.330	0.097	*p* > 0.05	0.485	0.106	*p* > 0.05
Rural	0.639	0.136		0.330	0.121		0.485	0.129	

**Table 4:** Average concentration of lead in hard tissues of impacted teeth (*μ*g/g).

Tissue	Enamel			Dentin			Total		
Place of residence	Concentration (*μ*g/g)	SD	*α* = 0.05	Concentration (*μ*g/g)	SD	*α* = 0.05	Concentration (*μ*g/g)	SD	*α* = 0.05
Urban	1.655	0.145	*p* = 0.0001	2.315	0.171	*p* = 0.0507	1.985	0.158	*p* = 0.0010
Rural	1.208	0.276		2.110	0.344		1.659	0.260	
